The article "Effect and Safety of ALA-PDT Combined with 1550 nm Fractional Therapy Laser in Treating Rosacea" was retracted in 2023. Reasons: signs of a paper mill; suspected computer-generated content; unreliable results or conclusions; concerns about the data.

# Effect and Safety of ALA-PDT Combined with 1550 nm Fractional Therapy Laser in Treating Rosacea

**DOI:** 10.1155/2022/3335074

**Published:** 2022-07-12

**Authors:** Hefei Wang, Xiaoxia An, Zhengli Wang

**Affiliations:** Heilongjiang Provincial Hospital, Harbin, Heilongjiang, China

## Abstract

**Objective:**

To explore the clinical effect and safety of 5-aminolevulinic acid photodynamic therapy (ALA-PDT) combined with 1550 nm fractional laser therapy in the treatment of rosacea.

**Methods:**

114 patients with type I and type II rosacea treated in our hospital from March 2018 to April 2020 were recruited. They were randomly assigned (1 : 1 : 1) to receive ALA-PDT (photodynamic group), 1550 nm fractional laser (laser group), or ALA-PDT and 1550 nm fractional laser therapy (combination group). Outcome measures included skin lesion scores, efficacy, and adverse reactions.

**Results:**

After treatment, patients in the three groups showed lower skin lesion scores than before treatment, and the combination group showed significantly lower results than the other groups (*P* < 0.05). There was no significant difference in the total efficacy among the three groups (*P* > 0.05), but the combination group outperformed the other groups in the comparison of the efficacy levels (*P* < 0.05). Edema with lupus erythematosus, pain, and burning sensation was found in some cases but disappeared within 2 to 4 days after symptomatic treatment without interference with subsequent treatment. No patients had pigmentation, hypopigmentation, scars, or other serious adverse reactions.

**Conclusion:**

In the treatment of rosacea, ALA-PDT combined with a 1550 nm fractional laser can reduce redness and facilitate skin remodeling, with high efficacy and safety, so it is worthy of clinical promotion and application.

## 1. Introduction

Rosacea is a common chronic inflammatory skin disease and is mostly found in people aged 30 to 50 years. It usually appears on the face, especially on the cheeks [1]. Rosacea is divided into telangiectasia rosacea (type I), papulopustular rosacea (type II), hyperplastic granulomatous rosacea (type III), and ocular rosacea (type IV), among which type I and type II are more common [2]. The disease seriously compromises the appearance of patients and leads to various degrees of physical and psychological stress. The onset of the disease may be related to vasoconstriction disorders, infection, diet, and mental stress. The treatment of rosacea includes oral medication, topical tacrolimus ointment, laser, and 95 nm pulsed dye laser, but efficacy is unfavorable [3, 4]. In recent years, the development and promotion of 5-aminolevulinic acid photodynamic therapy (ALA-PDT) have significantly ameliorated the treatment efficacy [5]. In traditional Chinese medicine, rosacea is described as “acne is caused by sweating and dampness” due to wind, dampness, heat, and insect toxicity. A prior study showed that ALA-PDT combined with Cuochuang Kangfu Decoction is a common method for rosacea [6]. The decoction is derived from the formula “Pipa Qingfei Decoction and Huanglian Jiebiao Decoction” under the guidance of traditional Chinese medicine theory. This formula integrates clinical experiences and is developed based on modern etiology and pharmacological research. The combination of all the herbs in the formula works to “clear heat and detoxify, cool the blood and subdue carbuncles, relieve depression, and disperse stasis.” Combination therapy is complementary to the strengths of multiple therapeutic regimens with simple operation, precise efficacy, and no increased bacterial resistance. In the past two years, our hospital had adopted the ALA-PDT combined with a 1550 nm fractional laser therapy for the treatment of type I and type II rosacea and achieved good efficacy.

## 2. Materials and Methods

### 2.1. General Materials

Patients with type I and type II rosacea in our hospital from March 2018 to April 2020 were recruited in this study. Inclusion criteria were as follows: ① patients who were diagnosed with type I and type II rosacea jointly by two physicians; the diagnostic criteria were based on the Pillsbury classification, grade II: acne and inflammatory papules; grade III: pustules in addition to acne and inflammatory papules; grade IV: nodules, cysts or scarring in addition to acne, inflammatory papules, and pustules, with grades II-III being moderate rosacea and grade IV being severe rosacea [2]; ② with complete data and age of 18 to 60 years; ③ without any treatment history of glucocorticoids, estrogen, and tretinoin in the past 30 days; and ④ patients who voluntarily participated in this study and provided written informed consent. Exclusion criteria were as follows: ① patients with a history of photosensitivity; ② with severe immune diseases; ③ with pregnancy, breastfeeding, or pregnancy plan in the past 3 months; ④ with laser treatment in the past 6 months; ⑤ with skin tumor; ⑥ with the withdrawal of consent; and ⑦ with a history of the systemic use of retinoid preparations within 6 months.

The study finally enrolled 114 patients with type I and type II rosacea, and they were randomly assigned a photodynamic group (*n* = 38), a laser group (*n* = 38), or a combination group (*n* = 38). This study was approved by the medical ethics committee of our hospital, and the number of ethics approval was 2017-11-19.

### 2.2. Methods

The photodynamic group was given ALA-PDT therapy. The aminolevulinic acid hydrochloride powder (Aila, manufacturer: Shanghai Fudan Zhangjiang Biomedical Co., Ltd., approval number: National Medicine Zhunzi 2007007, specification: 118 mg) and a temperature-sensitive hydrogel were mixed into 5% fresh gel and then applied evenly to the affected parts after cleansing face and wrapped with a shading paper for 2 hours. Then, the patients wearing protective glasses were treated with an LED photodynamic instrument manufactured by Wuhan Yage Optoelectronics Technology Co., Ltd., with an output wavelength of about 635 nm, continuous adjustment, and a power of 70–100 mW, and the distance of about 10 cm. The affected parts were irradiated for 20 minutes and given cold spray after irradiation, once a week, with 4 times in total. Sun exposure was prohibited during treatment.

The laser group received a 1550 nm fractional laser therapy. A Sellas-Evo produced by Daejeon Sellas in South Korea with a fixed model was used for treatment, with a pulse width of 0.48 ms, the frequency of 1500 Hz, the density of 100 PPA, the initial energy of 40–50 mJ, and the maximum energy of 45-85 mJ. Its cooling system was Smart CoolTM from Cynosure, USA. Before treatment, the target area was routinely disinfected and given lidocaine cream externally for anesthesia. The treatment was performed once every 3 weeks for 4 times. After treatment, patients were given a soothing mask to cold compress for half an hour, and sun exposure was prohibited within 7 days.

The combination group received the ALA-PDT combined with 1550 nm fractional laser therapy, once every 3 weeks, with 2 times in total. Sun exposure was prohibited within 7 days. After treatment, the patients were given a soothing mask to cold compress for half an hour, and sun exposure was prohibited within 7 days.

After returning home, the three groups of patients should pay attention to their diet, strengthen their nutrition, eat more fresh vegetables and fruits, not eat spicy and greasy, and irritating foods such as peppers, green onions, and ginger, coffee, alcohol, etc. And iodine-containing drugs and iodine-containing foods (e.g., kelp and shellfish) should be avoided since they might aggravate the disease [3]. During the recovery period, patients are required to avoid fatigue and nervousness, pay attention to rest, and avoid hot and cold stimuli such as hot baths, saunas, and prolonged exposure to the cold or hot sun that would result in pigmentation. Additionally, patients are should not use sunscreen within a week after treatment, only wear hats, and umbrellas to avoid sunlight. Moreover, patients should avoid strenuous exercise for a month, and clean their faces with warm water [3].

### 2.3. Observation Indicators

#### 2.3.1. Skin Lesion Score Evaluation

Two senior qualified physicians evaluated the facial erythema, telangiectasia, papules, impetigo, and itching, as shown in Table 1 [6]. The sum of points was the skin lesion score.

(1) $$\begin{array}{c} \text{efficacy index}=\frac{\left(\text{skin lesion score before treatment}-\text{skin lesion score after treatment}\right)}{\text{skin lesion score before treatment}}\times 100\%. \end{array}$$

#### 2.3.2. Efficacy Evaluation

The scoring investigators and patients were double-blind. The global physician's standards for the treatment of rosacea [7] were used to assess the efficacy. The efficacy index of 100% meant recovery, 75%–99% for significant efficacy, 50%–74% for improvement, and <50% for ineffectiveness. Effective rate = (recovery + significant efficacy)/cases × 100%. During the treatment and follow-up, adverse reactions were recorded, and patients with the withdrawal of consent due to adverse reactions or unsatisfactory efficacy were excluded.

### 2.4. Statistical Methods

In this study, the statistical software SPSS19.0 was used to process all the obtained data. The quantitative data were expressed as ($\bar{x}\pm s$), and analysis of variance was used for the comparison of data conforming to the normal distribution and equal variance among multiple groups. If differences were statistically significant, a pairwise comparison was performed. Dunnett-*t* test was used for pairwise comparisons, and if differences were not statistically significant through analysis of variance, no pairwise comparison was performed. The qualitative data were expressed as rates (%) and processed by the *χ*^2^ or rank-sum test, and rank data were tested with the rank-sum test. *P* < 0.05 indicated that the difference was statistically significant.

## 3. Results

### 3.1. Comparison of Baseline Data

There was no statistically significant difference in the baseline data (*P* > 0.05), as shown in Table 2.

### 3.2. Comparison of Skin Lesion Scores before and after Treatment

After treatment, patients in the three groups had lower skin lesion scores compared with those before treatment, and the combination group had significantly lower results than the other two groups (*P* < 0.05) (see Table 3).

### 3.3. Comparison of Efficacy

There was no statistically significant difference in the effective rate among the three groups (*P* > 0.05), but the combination group was significantly better in the comparison of efficacy among the three groups (*P* < 0.05) (see Table 4). The efficacy of the combination group before and after treatment is shown in Figure 1.

### 3.4. Comparison of Adverse Reactions

Edema with lupus erythematosus, pain, and burning sensation was found in some cases but disappeared within 2 to 4 days after symptomatic treatment without interference with subsequent treatment. No patients had pigmentation, hypopigmentation, scars, or other serious adverse reactions (see Table 5).

## 4. Discussion

Rosacea is one of the most common skin diseases characterized by inflammatory and noninflammatory lesions that may develop into scarring. Traditional rosacea treatment is challenged due to resistance to P. acnes, which necessitates new treatments [8]. Photodynamic therapy (PDT) is a photochemical reaction that uses photosensitizers to accumulate in tissues after entering the body and is excited under laser irradiation to generate reactive oxygen species, especially singlet oxygen, which in turn leads to cell damage and even death. At present, PDT has become the main treatment method in dermatology and has achieved promising results [8]. Recent molecular studies suggest that altered innate immune responses are involved in the pathogenesis of vascular and inflammatory diseases in patients with rosacea [9]. This study showed that PDT induces the formation of singlet oxygen production, resulting in the death of P. acnes. Studies also have shown that the pathogenesis may be related to the immune response caused by skin microorganisms [9, 10]. Among them, Demodex and *Staphylococcus* epidermidis are considered to be two common microorganisms. PDT can reduce the ability of staphylococcal biofilm and can eliminate Demodex mites, yielding a promising therapeutic effect on rosacea [10].

Studies have revealed an abnormal skin barrier function in patients with rosacea, characterized by a decrease in skin moisture and an increase in transepidermal water loss and pH. This disease is induced by internal and external factors, such as diet, tobacco and alcohol, drugs, climate, and emotions [8, 9]. Current treatment methods for rosacea include oral medicine, topical medicine, topical Chinese medicine, and pulsed laser, but the efficacy is mediocre [10]. As a new technology for the treatment of rosacea, ALA-PDT has attracted much attention in recent years and demonstrated considerable enrichments in the treatment efficacy of rosacea [11, 12]. ALA-PDT targets the exogenous 5-aminolevulinic acid (ALA) as a photosensitizer, acts specifically in the sebaceous gland unit, selectively destroys the sebaceous gland cells by the light of a specific wavelength, and inhibits the secretion of the sebaceous gland, only with reversible edema or mild inflammation in the epidermis and dermal cells [13]. Studies have found that the porphyrin secreted by propionibacterium acnes and ALA are absorbed by the sebaceous glands and then converted into protoporphyrin IX, and the singlet oxygen and free radicals are produced by which under the irradiation of specific light eliminate propionibacterium acnes [14]. In addition, ALA-PDT also improves the abnormal keratinization of sebaceous glands of hair follicles while exerting anti-inflammatory effects and boosting recovery [15].

1550 nm nonexfoliation fractional laser exerts a fractional photothermal effect, destroys the connection between the dermis layer and the epidermis, and forms subepidermal fissures. Moreover, its discontinuous matrix arrangement of microbeams results in less harm to the skin and facilitates the recovery of patients [16, 17]. In addition, nonexfoliation fractional laser activates various cytokines and related enzymes, promotes the remodeling of collagen fiber and dermis, and plays a role in scar restoration, photoaging reduction, and skin rejuvenation [18, 19]. In the present study, 1550 nm fractional laser therapy was used for the treatment of rosacea to kill local propionibacterium, improve the local microenvironment, and inhibit the secretion of sebaceous glands. In addition, 1550 nm fractional laser therapy destroys local capillaries, has a significant effect on telangiectasia rosacea, and prevents or reduces scars and adverse reactions to a certain extent.

Based on photodynamic therapy, 1550 nm fractional laser therapy is applied to evenly perform skin restoration and promote skin remodeling, which is considered a new method to achieve treatment [20, 21]. The results of this study showed that after treatment, patients in the three groups showed lower skin lesion scores than before treatment, and the combination group outperformed the other groups. There was no statistically significant difference in the effective rate among the three groups, but the combination group was significantly better in the efficacy levels. Cases of different degrees of edema with lupus erythematosus, pain, and burning sensation were found, but they disappeared within 2 to 4 days after symptomatic treatment and did not affect subsequent treatment. No patients in the three groups had pigmentation, hypopigmentation, scars, or other serious adverse reactions. In addition to a strong inhibition of photodynamic specificity on sebaceous gland secretion, 1550 nm fractional laser therapy compensates the shortcomings of photodynamic therapy, promotes the restoration and remodeling of epidermis and dermis, reduces damage to the skin, and boosts recovery. A key feature of rosacea is its high sensitivity to the external environment, for which a soothing mask was used as a cold compress and the patients are prevented from sunlight after treatment, which significantly reduces skin irritation. Postoperative nursing acted a pivotal part in recovery and postoperative sun protection. In contrast to systemic treatment with antibiotics, estrogen and progestin, and retinoic acid, which have resulted in increased bacterial resistance and various drug-related adverse effects, safe and effective physical treatments, such as ALA-PDT combined with 1550 nm fractional laser, have become a new trend in the treatment of rosacea.

## 5. Conclusion

ALA-PDT combined with 1550 nm fractional laser therapy can quickly mitigate redness and facilitate skin remodeling, with high efficacy and safety, so it was worthy of promotion and application in clinical practice. The small sample size and short observation time of this study might lead to biased results, so larger sample size and long-term follow-up are required for further investigation.

## Figures and Tables

**Figure 1:** Comparison of rosacea before and after treatment. (a) Before treatment in the combination group; (b) after the first treatment in the combination group; (c) after treatment in the combination group.

**Table 1:** Skin lesion score evaluation.

Score (points)	Erythema	Telangiectasias	Papule	Impetigo	Itch
0	No	No	No	No	No

1	Mild symptoms, mainly distributed in the middle of the face, or a few on the full face	Small blood vessels less than 0.2 mm in diameter, with an area less than 10% of the face	Small	Small	Mild

2	Obvious symptoms, mainly distributed in the middle of the face, or the entire face	More small blood vessels and (or) a few large blood vessels with a diameter greater than 0.2 mm, occupying 10%–30% of the face	Medium	Medium	Tolerable

3	Severe symptoms, widely distributed throughout the face	A large number of small blood vessels and (or) large blood vessels with an area larger than 30% of the face	Severe	Severe	Unbearable

**Table 2:** Comparison of baseline data.

Group	ALA-PDT group (*n* = 38)	Laser group (*n* = 38)	Combination group (*n* = 38)	*F*/*X*^2^	*P*
Gender					
Male	12	14	10		
Female	26	24	28	0.974	0.614
Age (years)	34.80 ± 10.20	37.06 ± 10.55	36.42 ± 11.05	0.458	0.634
Course (years)	2.40 ± 0.62	2.75 ± 0.70	2.56 ± 0.73	2.487	0.088

**Table 3:** Comparison of skin lesion scores before and after treatment.

Time	ALA-PDT group (*n* = 38)	Laser group (*n* = 38)	Combination group (*n* = 38)	*F*	*P*
Before treatment	9.46 ± 2.40	10.10 ± 2.32	9.88 ± 2.60	0.673	0.521
After treatment	4.05 ± 1.02	3.88 ± 1.10^*∗*^	2.30 ± 0.60^*∗*^^#^	40.677	<0.001
*t*	12.79	14.93	17.51		
*P*	<0.001	<0.001	<0.001		

*Note.* Comparison with the ALA-PDT group, ^*∗*^*P* < 0.05 comparison with the laser group, ^#^*P* < 0.05.

**Table 4:** Comparison of efficacy.

Index	ALA-PDT group (*n* = 38)	Laser group (*n* = 38)	Combination group (*n* = 38)	*X* ^2^	*P*
Recovery	10	13	20	6.532	0.038
Significant effectiveness	20	18	15		
Improvement	6	6	2		
Ineffectiveness	2	1	1		
Effective rate (%)	30 (78.95)	31 (88.57)	35 (92.11)	2.771	0.25

**Table 5:** Comparison of adverse reactions.

Index	ALA-PDT group (*n* = 38)	Laser group (*n* = 38)	Combination group (*n* = 38)	*X* ^2^	*P*
Edema with lupus erythematosus	5	2	3	1.535	0.464
Pain	5	4	4	0.174	0.917
Burning sensation	6	5	5	0.145	0.93
Pigmentation	0	0	0	—	—
Hypopigmentation	0	0	0	—	—
Scar	0	0	0	—	—

## Data Availability

The data used to support the findings of this study are available from the corresponding author upon request.
